# Antimicrobial Activity against Oral Pathogens Confirms the Use of *Musa paradisiaca* Fruit Stalk in Ethnodentistry

**DOI:** 10.1155/2021/8663210

**Published:** 2021-09-04

**Authors:** Ernest Owusu-Boadi, Mainprice Akuoko Essuman, Gabriel Mensah, Emmanuel Ayamba Ayimbissa, Alex Boye

**Affiliations:** Department of Medical Laboratory Science, School of Allied Health Sciences, College of Health and Allied Sciences, University of Cape Coast, Cape Coast, Ghana

## Abstract

**Background:**

Ethnodentistry is the use of indigenous oral cleansing agents such as plant parts by local folks not only to maintain oral hygiene but also to treat oral infections. Mostly, ethnodentistry is inspired by traditions and belief systems of local communities. *Musa paradisiaca* is extensively cultivated and used in many cultures for its nutritional and medicinal values. In Ghana, the fruit stalk of *Musa paradisiaca* is used as an oral cleansing agent to maintain oral hygiene; yet this folk claim remains to be ascertained scientifically.

**Objective:**

The study assessed the antibacterial and antifungal effects of three extract fractions (aqueous, ethanol, and ethyl acetate fractions) of *Musa paradisiaca* fruit stalk against *Lactobacillus acidophilus*, *Aggregatibacter actinomycetemcomitans*, and *Candida albicans*, common oral pathogens implicated in dental caries and periodontitis.

**Materials and Methods:**

Aqueous, ethanol, and ethyl acetate fractions of *Musa paradisiaca* fruit stalk were prepared by cold maceration and qualitatively screened for their phytochemical composition. Antimicrobial effects of the three extract fractions were assessed by using serial broth dilutions at increasing concentrations (62.5, 125, 250, 500, and 1000 *µ*g/ml) and compared to standard antimicrobial agents (erythromycin, doxycycline, and fluconazole). Subsequently, the absorbances of the microbial suspensions treated with increasing concentrations of the extract fractions were measured at 450 nm, and the cell densities were determined.

**Results:**

Except for the aqueous extract, which was less effective in decreasing microbial growth, the ethyl acetate and the ethanol extract fractions demonstrated antimicrobial efficacies comparable to those of the standard drugs. All three extract fractions demonstrated concentration-dependent growth inhibitory effects on the tested oral pathogens although not as effective as the standard drugs used.

**Conclusion:**

*Musa paradisiaca* fruit stalk has demonstrated antimicrobial effects against *Lactobacillus acidophilus*, *Aggregatibacter actinomycetemcomitans*, and *Candida albicans*, common oral pathogens implicated in dental caries and periodontitis, and this finding confirms in part folk use of *Musa paradisiaca* fruit stalk as a traditional dental care agent. Thus, the fruit stalk of *Musa paradisiaca* could be explored for use as a cheap and readily available dental care agent for people entrapped in the poverty line.

## 1. Introduction

Despite advancements in dentistry, oral diseases (dental caries, periodontitis, bleeding gums, toothache, oral sores, bad breath, tooth sensitivity, tooth loss, and oral cancer) remain a major health problem worldwide [1, 2]. Over 2.3 billion people are reported suffering from caries of permanent teeth and more than 530 million children are suffering from caries of primary teeth [3]. Evidence abounds linking risk of colorectal cancer, gum bleeding, toothache, preterm birth among pregnant mothers, chronic kidney disease, myocardial infarction, and stroke to oral diseases [4–9]. It is reported that most forms of periodontal diseases such as plaque, dental caries, halitosis, gingivitis, periodontitis, and toothache are caused by a complex and elusive activity of over 600 polymicrobial species inhabiting the oral cavity [10]. Common among these oral pathobionts are Gram-positive and -negative bacteria such as *Veillonella* species, *Atopobium* species, *Prevotella* species, *Streptococcus mutans*, *Lactobacillus* species, *Enterococcus faecalis* and some nonmutant streptococci, which are associated with caries formation and progression [10–12]. Also, common Gram-negative bacteria, such as *Aggregatibacter actinomycetemcomitans*, have been associated with aggressive periodontitis [13], while commensal yeasts, such as *Candida albicans*, are also implicated in oral candidiasis [14], requiring holistic treatments.

Treatment of oral diseases involves the use of various agents having demonstrable antimicrobial, antioxidant, anti-inflammatory, antifungal, and analgesic effects. Risk of urticaria, taste masking, increased calculus formation, stained teeth and mucous membranes, oral mucosa desquamation, and parotid swelling are associated with long-term use of some conventional oral care agents, such as chlorhexidine [11, 15, 16]. Given the incidence of oral disease, increased microbial resistance, adverse effects associated with some conventional oral care agents currently used in oral care, and the high cost of these conventional oral care agents, it has become necessary to prospect for alternatives treatments which are relatively cheaper, readily available, effective, and safe.

Use of plants and plant-derived products to improve human health has been in existence for centuries even before the dawn of modern medicine. Most of the curative effects of medicinal plants have been determined over hundreds of years through centuries of uneventful use [17, 18]. The World Health Organization (WHO) has reported that in developing countries, 65–80% of populations depend on traditional therapies, mostly plant-based therapies [17]. Thus, the WHO has recommended that countries should formulate national policies and regulations to integrate plant-based therapies into their healthcare systems [19].

Interestingly, use of plant-based therapies to improve general health is quite common in Ghana [20]. For instance, *Musa paradisiaca* fruit stalk is commonly used in rural Ghana to maintain oral hygiene; however, this folk claim remains to be ascertained scientifically. Ecologically, *M. paradisiaca* (family, Musaceae) is distributed in the tropical and subtropical regions of the world. Traditionally, *Musa paradisiaca* is used for treatment of diarrhea, dysentery, intestinal lesions in ulcerative colitis, diabetes, in sprue, uremia, nephritis, gout, hypertension, and cardiac disease [21, 22]. In view of the ethnobotanical importance of *M. paradisiaca*, many studies have investigated some of its traditional uses. For example, the peels of the fruit have demonstrated antifungal activity against *C. albicans* [23]. Extracts of unripe fruit peels and leaves of *Musa paradisiaca* have demonstrated antimicrobial activity against *Pseudomonas* species, *Staphylococcus aureus, Escherichia coli*, and *Proteus mirabilis* [23, 24]. Also, extracts from various parts of *M. paradisiaca* have demonstrated antidiarrheal, hypoglycemic, antioxidant, antihypertensive, wound healing, antiallergic, antimalarial, leishmanicidal, and anti-snake venom activities [21, 25, 26]. The observed pharmacological properties were attributed to organic and inorganic components of *M. paradisiaca* including vitamins, lutein, carotene, potassium, and magnesium [23, 27] as well as phytochemicals such as flavonoids, serotonin, tryptophan, indole, tannins, and triterpenes [21, 22]. The present study assessed the antimicrobial effect of *M. paradisiaca* fruit stalk extracts against three common oral pathogens implicated in dental caries and periodontitis.

## 2. Materials and Methods

### 2.1. Chemicals and Reagents

The materials used in the study included Sabouraud Dextrose agar (SDA), peptone water, blood agar, doxycycline (Actavis, Barnstaple, UK), erythromycin (Concordia International, Capital House, UK), and fluconazole (FDC International, Fareham Harts, UK). Also, ethyl acetate, ethanol, sodium hydroxide (VWR Prolab Chemicals, France), hydrogen peroxide, Wagner's reagent, Mayer's reagent, and ferric chloride chemicals used were of analytical grade. Equipment such as a gas bath oscillator, dry-air oven, aerobic incubator, and other apparatus such as Petri dishes, beakers, and pipettes were also used.

### 2.2. Plant Collection, Identification, and Authentication

Fresh *M. paradisiaca* fruit stalks (red arrows in Figure 1) were collected from Abura market in the Cape Coast Metropolis, Ghana. Identification and authentication were done by Mr. Francis Otoo, the curator at the Herbarium Unit, School of Biological Sciences, University of Cape Coast. The green outer coverings of the fruit stalk were removed with a clean sharp knife and discarded. The remains were then chopped into small pieces and shade dried for two weeks. The dried fruit stalk remains were pulverized manually by pounding with mortar and pestle. The powdered samples were packed into transparent plastic sample bags, labeled, and stored at room temperature.

### 2.3. Preparation of *Musa paradisiaca* Fruit Stalk Extracts

Three flat-bottomed flasks were each filled with 20 g of the powdered sample. A 200 ml each of distilled water, ethanol, and ethyl acetate were added to each of the flasks and appropriately labeled. The flasks were corked with clean cotton wool and aluminum foil and allowed to stand with intermittent shaking on a mechanical shaker for 72 hours. After shaking, all four samples were vacuum filtered through filter paper (Whatman No. 54) separately with a Buckner funnel and a suction pump. The filtrates were each collected into separate conical flasks and labeled. The four samples were then concentrated using a rotary evaporator and the concentrates transferred into weighed and labeled crucibles for further evaporation on a water bath. All four samples were then placed into a desiccator and allowed to dry. The resultant fractions were weighed and labeled according to the solvent used to extract them as aqueous (AEMP), ethanol (EEMP), and ethyl acetate fractions (EAMP). Five different concentrations (62.5, 125, 250, 500, and 1000 *µ*g/ml) were prepared from each of the extracts by serial dilution.

### 2.4. Preliminary Phytochemical Screening

The phytochemicals screened for included alkaloids, flavonoids, tannins, terpenoids, saponins, and phenols as follows.

#### 2.4.1. Test for Alkaloids

Presence of alkaloids was determined as previously described [28]. Briefly, 0.4 g of the dried extracts was dissolved in 5 ml of 1% HCl and the mixture warmed and filtered. 1 ml of filtrate was treated separately with (a) a few drops of potassium mercuric iodide (Mayer's reagent) and (b) potassium bismuth (Dragendorff's reagent). Turbidity or precipitation with either of these reagents was taken as evidence for the existence of alkaloids.

#### 2.4.2. Test for Flavonoids

The presence of flavonoids was assessed by using a previously described method. Briefly, 0.5 g of each extract fraction was suspended in 1 ml of distilled water stirred and filtered to obtain a filtrate. A 0.5 ml of dilute ammonia solution was added to 0.5 ml of the filtrate followed by the addition of few drops of concentrated sulphuric acid. Appearance of yellow coloration confirmed the presence of flavonoids.

#### 2.4.3. Test for Tannins

Tannins were detected using a modified version of the Ferric chloride test as described previously [28]. Briefly, 2 drops of 1% aqueous ferric chloride reagent were added to 0.5 ml of crude extract and observed for the formation of blue-black or green coloration, which indicated the presence of tannins.

#### 2.4.4. Test for Phenolic Compounds

Phenolic compounds were detected using a modified version of the Folin–Ciocalteu procedure [29]. Briefly, 200 *μ*l of crude extract was added to 2 ml of 3% aqueous sodium carbonate, followed by the addition of 200 *μ*l Folin–Ciocalteu reagent. The mixture was allowed to stand for 30 minutes at room temperature. The formation of blue/gray colour indicated the presence of phenolic groups.

#### 2.4.5. Test for Triterpenoids

Triterpenoids were detected using a modified version of the Salkowski test [30]. Briefly, 1 ml of extract was slowly added to 400 *µ*l chloroform, followed by the careful addition of 400 *µ*l concentrated sulphuric acid. Formation of a red/brown/purple colour at the interface indicated the presence of triterpenoids.

#### 2.4.6. Test for Cardiac Glycosides

Cardiac glycosides were detected using a modified version of the Keller–Kiliani test [29]. 500 *μ*l of extract was added to 500 *μ*l glacial acetic acid. A few drops of 1% aqueous iron chloride and concentrated sulphuric acid were then carefully added. The presence of a red/brown ring of the interface indicated deoxy sugar characteristic of cardiac glycosides.

#### 2.4.7. Test for Anthraquinones

Anthraquinones were detected using modified versions of the Kumar and Ajaiyeoba tests [28, 29]. The modified Kumar test involved the addition of a few drops of concentrated sulphuric acid to 500 *μ*l pure extract, followed by the careful addition of 500 *μ*l of ammonia. A rose-pink colour indicated the presence of free anthraquinones. For the Ajaiyeoba test, 450 *μ*l of crude extract was added to 50 *μ*l concentrated HCl and allowed to stand at room temperature for several minutes. 500 *μ*l of chloroform was then carefully added. The formation of a rose-pink colour indicated the presence of free hydroxyl anthraquinones.

### 2.5. Ethical Clearance

The study was approved (UCCIRB/CHAS/2016/29) by the University of Cape Coast Institutional Review Board (UCCIRB) and the management of University of Cape Coast Dental Clinic. Also, patients' consent was sought for by means of a verbal or written agreement after the aim of the study was clearly explained to the patients.

### 2.6. Acquisition, Culturing, and Identification of Test Organisms

This was a laboratory experimental study to determine the antibacterial and antifungal activities of aqueous, ethanol, and ethyl acetate extracts of *Musa paradisiaca* fruit stalk against three common oral pathogens. The test bacteria were acquired from the Dental Clinic of University of Cape Coast. The research was carried out in the laboratories at the Department of Medical Laboratory Science, University of Cape Coast and Cape Coast Teaching Hospital. The plant extracts were screened for phytochemicals present and then assayed for the antibacterial activity using serial broth dilution. Test fungal strains, *Candida albicans*, that were used in the study are clinical isolates and were provided by the Microbiology Laboratory of Cape Coast Teaching hospital. These species were cultured on Sabouraud Dextrose agar (SDA) plates and incubated at room temperature (28 ± 3°C) for 3 days. *Candida* species were subcultured unto SDA supplemented with chloramphenicol and incubated at 37°C for 72 hours to obtain pure isolates. Identification of *Candida albicans* was done using germ tube test. Bacterial strains, *Lactobacillus acidophilus* and *Aggregatibacter actinomycetemcomitans*, were obtained by taking dental swabs from the patients who visited the University of Cape Coast Dental Clinic. Using sterile cotton swab sticks, swabs were taken from deep cavities in the teeth and also from plaques on the teeth. The swabs were placed in Bijou bottles containing sterile peptone water and incubated overnight at 35°C. Bacterial colonies were subcultured on blood agar and incubated at 35°C for 24 hours. After incubation, colony appearance, biochemical tests as previously performed [31], and Gram staining to confirm the presence of *Lactobacillus acidophilus* and *Aggregatibacter actinomycetemcomitans* were performed.  Table 1 shows a summary of results of biochemical tests that were conducted to confirm or otherwise the identity of the test organisms.

### 2.7. Serial Broth Dilution

Each fraction of the extract was dissolved in sterile distilled water to form stock concentrations of 10380 *µ*g/ml, 10230 *µ*g/ml, and 10300 *µ*g/ml for ethanol, aqueous, and ethyl acetate fractions, respectively. From these stock solutions, working concentrations of 1000, 500, 250, 125, and 62.5 *µ*g/ml were prepared and used for the tests for antimicrobial activity. Fluconazole (FDC International, Fareham Harts, UK), doxycycline (Actavis, Barnstaple, UK), and erythromycin (Concordia International, Capital House, UK) were used as positive control drugs for *Candida albicans*, *Aggregatibacter actinomycetemcomitans*, and *Lactobacillus acidophilus*, respectively, with the same concentration as the fractions. A 0.5 McFarland standard was used to standardize each of the three freshly cultured isolates to a density of 1.5 × 10^8^ CFU/ml in sterile peptone water. 0.5 ml of this inoculum was added to sterile test tubes with the label of the fraction and the concentration. 1 ml of each concentration of the fractions was added to the corresponding test tubes containing the inoculum. The same was done for the drug control with the drug replacing the fractions instead. Turbidity standard for the bacteria was prepared by adding 0.5 ml of the inoculum to 1 ml of sterile peptone water whereas sterility standard was prepared by using sterile peptone without any additions. Bacterial and fungal suspensions were incubated at 35°C and 25°C, respectively, for 24 hours. Absorbance of the content of each of the test tubes was determined at a wavelength of 450 nm. The density of each suspension after incubation was determined by proportion as it was compared to the density and absorbance of the 0.5 McFarland. Each experiment was repeated at least three times.

### 2.8. Statistical Analysis

Data generated from the antibacterial effect of the three plant extracts of *Musa paradisiaca* on the 2 test bacteria and 1 fungi specie were entered and organized in Microsoft Excel. These data were then exported to IBM SPSS version 24.0 (SPSS Inc., Chicago, IL, USA) to compute descriptive statistics of the mean and standard deviations. Data were also analyzed with GraphPad Prism version 6 (GraphPad Software, San Diego, CA, USA) to perform one-way analysis of variance (ANOVA) using Tukey's multiple comparisons to compare between different antibacterial activities of different extract concentrations against each test bacteria versus controls. Two-way ANOVA was used to determine if there were significant differences in the antibacterial activities between the aqueous, ethanol, and ethyl acetate extracts at varying concentrations against the test bacteria. *P* values ≤ 0.05 were considered statistically significant in all analyses.

## 3. Results

### 3.1. Yield of Extracts and Phytochemical Screening

The aqueous extract yielded the highest fraction of crude extract of *M. paradisiaca* stalk. Upon phytochemical screening of *M. paradisiaca* fruit stalk extracts (MPFSEs), it was observed that phenols were present in all the three extracts fractions (Table 2). Triterpenoids and cardiac glycosides were detected in the ethyl acetate fraction. All fractions except the aqueous fractions showed presence of alkaloids (Table 2).

### 3.2. Effect of Extracts on Mean Cell Density (CFU/mL) of *L. acidophilus*

Erythromycin demonstrated concentration-dependent decrease in mean cell density of *L. acidophilus.* Although the extracts fractions demonstrated inhibitory effects on mean cell density of *L. acidophilus*, this was not comparable to that of erythromycin (Figure 2). Among the three extract fractions, the ethyl acetate fraction demonstrated significant inhibitory effects on cell density, and this inhibitory effect was concentration dependent.

### 3.3. Effect of Extracts on Mean Cell Density (CFU m/L) of *A. actinomycetemcomitans*

Both doxycycline, aqueous and ethanol fractions did not demonstrate significant inhibitory effects on mean cell density of *A. actinomycetemcomitans*. The ethyl acetate fraction demonstrated concentration-dependent inhibitory effect on mean cell density (Figure 3).

### 3.4. Effect of Extracts on Mean Cell Density (CFU m/L) of *Candida albicans*

Aqueous fractions of the extract had no inhibitory effect on mean cell density of *C. albicans* compared to that of fluconazole. Ethyl acetate and ethanol fractions of the extract demonstrated concentration-dependent inhibitory effects on the mean cell density of *C. albicans* comparable to that of fluconazole (Figure 4). At the highest equipotent concentrations, the ethyl acetate fraction demonstrated more inhibitory potency than fluconazole (Figure 4).

### 3.5. Effect of Extracts on Growth of Test Organisms

All the three fractions (aqueous, ethanol, and ethyl acetate) demonstrated some degree of growth inhibition against the three test organisms (*L. acidophilus, A. actinomycetemcomitans*, and *C. albicans*). Among the fractions, ethyl acetate fraction was the most potent against all the test organisms (Figure 5).

## 4. Discussion

This study has demonstrated that extracts from *M. paradisiaca* fruit stalk have antimicrobial effects against common oral pathogens (*Lactobacillus acidophilus*, *Aggregatibacter actinomycetemcomitans*, and *Candida albicans*), mostly implicated in oral infections. For instance, these pathobionts have long been linked to the initiation and progression of dental caries, oral thrush, and periodontitis [12, 14, 32]. Antimicrobial property is considered as one of the key hallmarks of oral care agents, in view of the involvement of pathogenic bacteria and fungal species in oral infections. The fruit stalk of *Musa paradisiaca* is used in rural Ghana to maintain oral hygiene. Specifically, a pulverized preparation of the fruit stalk of *Musa paradisiaca* with or without charcoal is used to clean the teeth and also to maintain oral hygiene. Use of *M. paradisiaca* fruit stalk by rural folks has been handed down many generations, and this age-old practice has been uneventful. At a time, that use of conventional oral cleansing agents has not only received a backlash for claimed adverse effects but also has been seen as expensive yet ineffective; it is refreshing to learn of readily available alternative or complementary oral care therapies. However, such alternative oral care therapies need to be verified scientifically to substantiate these claims.

In this study, three (aqueous, ethanol, and ethyl acetate) extract fractions of *M. paradisiaca* produced concentration-dependent inhibition of growth of the test oral pathogens; in particular, the ethyl acetate extract fraction demonstrated significant antimicrobial activity compared to the other extract fractions. Except for the aqueous extract, which did not demonstrate significant decrease in cell density of the test pathogens, the ethyl acetate and ethanol fractions demonstrated significant antimicrobial activity. The ethyl acetate extract demonstrated concentration-dependent broad-spectrum decrease in cell densities of the three test pathogens. In the case of the ethanol extract, antifungal activity against *Candida albicans* was observed. The current observed antimicrobial activity of *M. paradisiaca* fruit stalk extracts against oral pathogens implicated in oral infections complements that of other studies which showed that extracts from fruits, florets, root, leaves, and peels of *M. paradisiaca* possess antimicrobial properties [23, 27, 33, 34]. The current observation together with that of previous studies which demonstrated that *M. paradisiaca* has antimicrobial activity against *A. actinomycetemcomitans* [35] and *C. albicans* [23] clearly shows the possible prospects of *M. paradisiaca* as an alternative or complementary oral therapy that can be exploited for use by indigenous people.

The bioactivity of medicinal plants has always been linked to their phytochemical composition and functional group enrichment [36]. Antioxidant, antiproliferative, chemopreventive, and antimicrobial properties demonstrated by synergistic interactions of naturally occurring phytocompounds including alkaloids, phenolic compounds, tannins, saponins, and terpenoids have been reported in oral health [16, 37]. The present study showed that *Musa paradisiaca* fruit stalk contains alkaloids, terpenoids, cardiac glycosides, and phenols, which corroborates earlier reports on *Musa paradisiaca* [21, 23] and these phytocompounds possibly may account for the observed antimicrobial activity in the current study.

In increasing order, the antimicrobial activity of the three extract fractions of *M. paradisiaca* fruit stalk was in the order aqueous < ethanol < ethyl acetate, and this order of antimicrobial activity reflected their phytochemical composition and probably solvent system dependent. It was not surprising to observe that ethyl acetate fraction demonstrated significant antimicrobial activity as it extracted most of the phytocompounds, including alkaloids and cardiac glycosides, which were absent in the aqueous fraction (Table 2). Cardiac glycosides from other medicinal plants have demonstrated antifungal properties [38]. Thus, it is also possible that the antifungal activity demonstrated by the ethyl acetate and ethanol extract fractions of *M. paradisiaca* fruit stalk could be due to their cardiac glycoside components. Surprisingly, alkaloids and cardiac glycosides were absent in the aqueous extract fraction of *M. paradisiaca* fruit stalk in the current study. However, in a study involving fruit peel of *M. sapientum*, it was shown that the aqueous fraction demonstrated significant antibacterial effect compared to that of absolute ethanol fraction and this was linked to its alkaloidal components [39] and this observation stands at variance with the current observation where the aqueous fraction of *M. paradisiaca* fruit stalk demonstrated the least antimicrobial activity. In summary, the observed antimicrobial activity of the fractions (aqueous, ethanol, and ethyl acetate) directly relates to their ability to extract diverse compounds from the fruit stalk; however, disparity between the current results and that of other species in the genus *Musa* could be due to the differences in both species and the part of plant investigated.

## 5. Conclusion

*M. paradisiaca* fruit stalk extracts have demonstrated antimicrobial effects against *Lactobacillus acidophilus, Aggregatibacter actinomycetemcomitans*, and *Candida albicans*, and this observation perhaps adds credence to its folk use in maintaining oral hygiene. The observed antimicrobial activity is attributable to the phytochemical composition of *M. paradisiaca* fruit stalk; therefore, future studies should focus on bio-assay guided extraction, identification, and purification of specific antimicrobial phytocompounds with specific antimicrobial activity against oral pathogens.

## Figures and Tables

**Figure 1:** Areal part of *Musa paradisiaca* (plantain) showing fruit stalk (red arrow) and fruits.

**Figure 2:** Effect of extracts on microbial cell density of *Lactobacillus acidophilus*. Each bar is the mean cell density ± SD, *n* = 3.

**Figure 3:** Effect of extracts on microbial cell density of *A. actinomycetemcomitans*. Each bar is the mean cell density ± SD, *n* = 3.

**Figure 4:** Effect of extracts on microbial cell density of *C. albicans*. Each bar is the mean cell density ± SD, *n* = 3.

**Figure 5:** Inhibitory effects of extract fractions of *M. paradisiaca* fruit stalk on the of growth of (a) *Lactobacillus acidophilus*, (b) *Aggregatibacter actinomycetemcomitans*, and (c) *Candida albicans*.

**Table 1:** Results of biochemical tests to confirm *Lactobacillus acidophilus* and *Aggregatibacter actinomycetemcomitans*.

Test	Reaction
*Lactobacillus acidophilus*	
Gram reaction	+
2% NaCl tolerance	+
2% bile tolerance	+
Glucose fermentation	+
Galactose	+
Sucrose	+
Lactose	+
Mannose	+
Catalase	−
Motility	−
Indole	−
TSI	−
Citrate	−

*Aggregatibacter actinomycetemcomitans*	
Gram reaction	−
Glucose fermentation	+
Motility	−
Fructose	+
Maltose	+
Indole	−
Catalase	+
Oxidase	−

(+) indicates positive reaction; (−) indicates negative reaction.

**Table 2:** Percentage yield and qualitative phytochemical profile of the three extract fractions of *Musa paradisiaca* fruit stalk.

	Solvents for extraction		
	Aqueous	Ethanol	Ethyl acetate
Yield^*∗*^*N* (%)	1.82 (9.10)	0.53 (2.65)	0.24 (1.20)
Phytochemicals			
Phenols	+	+	+
Flavonoids	−	−	−
Anthraquinones	−	−	−
Tannins	−	−	−
Triterpenoids	+	−	+
Alkaloids	−	−	+
Cardiac glycosides	−	+	+

+ = present; − = absent; and ^*∗*^*N*/*Y* × 100, where *N* = mass of the extract and *Y* = mass of dry powdered fruit stalk (20 g).

## Data Availability

All data used to support the findings of this study are available within the article.
